# Face Recognition Algorithm Based on Multiscale Feature Fusion Network

**DOI:** 10.1155/2022/5810723

**Published:** 2022-03-18

**Authors:** Yunquan Li, Meizhen Gao

**Affiliations:** School of Information Engineering, Jiaozuo Normal College, Jiaozuo 454000, China

## Abstract

A face recognition model based on a multiscale feature fusion network is constructed, aiming to make full use of the characteristics of face and to improve the accuracy of face recognition. In addition, three different scale networks are designed to extract global features of faces. Multiscale cross-layer bilinear features of multiple networks are integrated via introducing a hierarchical bilinear pooling layer. By capturing some of the feature relationships between different levels, the model's ability to extract and distinguish subtle facial features is enhanced. Simultaneously, this study uses layer-by-layer deconvolution to fuse multilayer feature information, to solve the problem of losing some key features when extracting features from multilayer convolutional layers and pooled layers. The experimental results show that compared with the recognition accuracy of traditional algorithms, the recognition accuracy of the algorithm on Yale, AR, and ORL face databases is significantly improved.

## 1. Introduction

In recent years, face recognition has been widely used because of its stability, noncontact, and easy access. However, the complexity and changeability of the actual application scene environment, especially the changes in lighting, expression, occlusion, posture, and so on, will significantly affect the performance of face recognition.

Face recognition mainly consists of face detection, face representation, face matching, and other links. Face representation mainly includes feature extraction and feature dimensionality reduction. Feature extraction is the extraction of facial features that can reflect the identity of a specific face from the attribute elements of the face, thus becoming the key to the recognition of the entire face. The research of feature extraction is mainly divided into two categories: local feature extraction and global feature extraction. Global features focus on global properties, and classical methods include principal component analysis (PCA) [1] and linear discriminant analysis (LDA) [2]. Global features can reflect rough information, but cannot portray face details, which has great limitations when applied. The local feature-based method focuses on the micro-texture structure of the image, and the original image is encoded in a pattern to obtain a new feature image. It can maintain better stability for interference such as lighting and expression, which has been widely studied in recent years. At present, the methods of local feature extraction are mainly divided into two categories. One is local feature extraction methods based on manually designed descriptors, such as local directional number pattern (LDN) [3] and compressive binary pattern (CBP) [4]. It relies on the designer's prior knowledge to carefully design the code and calculate quickly with good results. Another type of local feature extraction method is based on learning descriptors, such as compact binary face descriptor (CBFD) [5] and context-aware local binary feature learning (CA-LBFL) [6]. It optimizes coding methods through unsupervised or supervised learning. Compared with manual descriptors, it uses pixel information with a larger sampling range to automatically encode, without the need to manually design specific encoding rules. However, this kind of method requires multiple iterations to find the optimal code, which is time-consuming and inefficient to calculate. The methods based on hand-designed descriptors have fast calculation speeds and good recognition performance, so they have been widely studied in recent years.

The literature [7] proposed that a local binary pattern (LBP) is a classical method for local feature extraction. It focuses on the local texture of the image and uses the local area information to replace the information of a single pixel, which has a good texture description ability, but LBP only uses grayscale information and abandons non-strength information, and there are many areas for improvement. The local direction number (LDN) pattern was proposed to overcome some of the drawbacks of methods such as LBP. It records the two directions where the edges respond strongest and weakest, capturing the main texture. However, the LDN only extracts gradient information based on the original edge response value, and the feature information is small. The literature [8] proposed a local directional texture pattern (LDTP) based on retaining the LDN edge response information, which enriched the gradient information by distinguishing the grayscale differences in the main directions, but ignored the extraction of the grayscale spatial information. The literature [9] proposed the gradient center symmetric local directional pattern (GCSLDP), which uses the difference in the edge response of the central symmetry point and the adjacent point to describe the face information and extracts the deeper gradient information, but ignores the texture details contained in the original edge response and does not accurately restore the face features. The literature [10] proposed a double-space local directional pattern (DSLDP), which preserves both the original edge response information and the edge response difference information of adjacent points. However, it only relies on marginal response operators to supplement gradient information, ignores the difference and intensity information of grayscale space, and cannot fully extract face features with strong differentiation. Both gradient information and grayscale information for an image are important components that describe the details of an image. The LBP method captures the grayscale information of the image, but ignores the gradient information that has a stronger ability to portray the edge details. Most of the LDN-like methods obtain gradient information based on edge response operators and lack effective utilization of grayscale information.

To solve the above problems, this study constructs an identification model based on multiscale bilinear pooled convolutional neural network. The recognition model has the following innovations: first, it designs and trains three coarse-scale networks applied to the classification of face features. The second is to use hierarchical bilinear pooling to capture the multiscale features of different networks and to explore the ability of neural networks to distinguish subtle changes in key areas of facial expressions such as mouth, eyebrows, and eyes. The third is to propose a multilayer information fusion method to obtain useful low-frequency information, thereby improving the performance of face classification.

This study consists of four main parts, namely the introduction of the first section, the convolutional neural network model in the second section, the experiment and analysis in the third section, and the conclusion in the fourth section, with the abstract and reference section.

## 2. The Proposed Algorithm

### 2.1. Neural Network Structure

This study proposes a multiscale hierarchical bilinear pooling network (MHBP) model, as shown in Figure 1. The 3-column network uses different convolutional-scale nuclei, *3, 5,* and *7,* respectively, to extract more elaborate facial features. Each column network has 9 convolutional layers and *3* maximum pooled layers. The same face image is input into a 3-column network, and the feature diagram of the last *3* convolutional layers of the same depth position is integrated into the feature map of the last *3* convolutional layers through the hierarchical two-line pooling layer, and the partial connections between different levels are captured to facilitate the classification of subsequent face features. It is not suitable for direct classification in that the integrated feature dimension is too high and there are many redundant features. Therefore, two layers of fully connected layer filter features need to be added to achieve face classification. The feature diagram in the figure is a brief schematic diagram of the feature map output of the last convolutional layer of the network, and the other layers are ignored, and the specific interaction mechanism is shown in Section 2.3.2.

To make better use of the different scale characteristics of the backbone network, this study proposes a multiscale attention interaction module, as shown in Figure 2.

The module first fuses the feature maps f3, f5, and f7 of the three coarse and fine-scale networks through 3 ×3, and one branch is activated by the sigmoid function [11]. After generating the feature weights, they are multiplied with the elements of the feature diagrams f3, f5, and f7, respectively, to obtain a rescaled feature map. Finally, the fusion feature elements activated by the parametric rectified linear unit (PReLU) function [12] are added to obtain the final respective outputs. Based on back propagation, the module is self-updating and learning, automatically selecting multiscale features that each branch needs to be fused. In this network training test, the module is added to the position between the two convolutional layers before the first three pooling layers of the network, and a total of 3 are added.

### 2.2. Model Parameter Configuration

The specific parameter configurations of the MHBP model are shown in Table 1 and Table 2. Table 1 and Table 2 omit the backbone network multiscale feature fusion module. According to the different resolutions of the output feature map, it can be divided into four stages. Each network has 2 convolutions in the first *3* stages and *3* convolutions in the latter stage. The *3* networks have a grayscale map of the common input of *48×48* sized facial images. The convolutional kernel sizes of the *3×3*，*5×5*，and *7×7* networks are *3×3, 5×5, and 7×7*, respectively, with 1 step size and padding and *32* convolutional kernels. *(3,2,1)* in Maxpool indicates that the filter size is *3×3*, the step size is *2*, and the fill is *1*. The output feature plot is *h×w×c*. Thereinto, *h* and *w* are the height and width of the feature map, respectively. *c* is the number of feature maps, that is the number of convolutional kernels. *18* sets of 512-dimensional face bilinear feature vectors are integrated through bilinear pooling. To avoid overfitting of the model, the accuracy of face image classification is further improved by improving the generalization ability of the model [13]. After each pooling layer, the dropout network is joined with a drop probability of *0.1*. Similarly, in the convergence classification stage, batch normalization (BN) and dropout networks are added after the *2* fully connected layers, where the probability of dropout networks is *0.5*. The goal is to enhance the network's ability to mine hidden features and thus improve model performance. The first fully connected layer is fully connected to *1024* neurons, while the second fully connected layer is fully connected to *512* neurons. The output layer is a softmax layer of *7* neurons that predicts the output of *7* faces.

### 2.3. Hierarchical Bilinear Pooling

Hierarchical bilinear pooling [14] interactive modeling of local pairwise features has proven to be a powerful tool for solving fine-grained recognition problems. To obtain a better face feature, a face mining method in the background of fine-grained recognition task is proposed. Through interactive modeling in different cross-layers, the middle layer features of different convolutional layers of the same scale network and different scale networks are integrated to achieve face recognition.

#### 2.3.1. Working Principle

The hierarchical bilinear pooling model is built based on the decomposition bilinear pooling model [15]. The process of factorization bilinear pooling is that the feature map extracted by the thickness scale trunk network is recorded as *I* *∈* *R*^*h×w×c*^, where *h*, *w*, and *c* are the height, width, and number of channels of the feature map, respectively. Let *i* *=* *[i*_*1*_*,i*_*2*_*,⋯,i*_*c*_*]*^*T*^ be a spatial position c-dimensional descriptor on *I*. Bilinear models are defined as follows:

(1) $$\begin{array}{c} k_{x}=i^{N}M_{x}i, \end{array}$$

where *k*_*x*_ is the output of a bilinear model. *M*_*x*_ *∈* *R*^*c×c*^ is the projection matrix. The bilinear model decomposes *M*_*x*_ into low-order outer product operations to obtain output features.

(2) $$\begin{array}{c} k=U^{N}\left(P^{N}i\circ Q^{N}i\right). \end{array}$$

*U* *∈* *R*^*d×o*^ is the classification matrix. *d* is the hyperparameter that determines the embedded dimension. *o* is the total number of image classification categories. *P* *∈* *R*^*c×d*^ and *Q* *∈* *R*^*c×d*^ are projection matrices for obtaining d-dimensional pooled eigenvectors from c-dimensional eigenvectors.

Bilinear pooling captures pairwise representation relationships and is an important technique for fine-grained recognition. The key areas for judging the face attributes of the face are only the areas near the eyes, eyebrows, nose, and the corners of the mouth, which is a fine work. This can therefore be done with the help of bilinear pooling. However, if you only focus on a single convolutional layer and completely ignore the cross-layer interaction of information, it will lead to the poor classification of face. This is because the activation of a single convolutional layer is incomplete, and each feature has multiple attributes, such as the shape of the mouth and the curvature of the corners of the mouth, which are essential for subtle changes in the face. Interlayer feature interactions between different convolutional layers can help capture the distinguishing features of subtle face. The use of cross-layer bilinear pools integrates more intermediate convolutional layers to further enhance the representation of face features. Features from different convolutional layers are extended to high-dimensional spaces through independent linear mappings (1×1 convolutions). The output face that integrates different cross-layer face features is as follows:

(3) $$\begin{array}{c} O_{o}=U^{N}concat\left(P^{N}i\circ Q^{N}j，P^{N}i\circ S^{N}k，Q^{N}j\circ S^{N}k，\cdots \right). \end{array}$$

*P ∈ R^c×d^*, *Q ∈ R^c×d^*, and *S ∈ R^c×d^* are, respectively, the projection matrices of interactive cross-layer convolution layer features *i*, *j* and *k*. The aggregated emoticon features from different cross-layers are fed into the fully connected layer and the softmax classification, and the softmax classification loss function is defined as follows:

(4) $$\begin{array}{c} L_{softmax}=-\frac{1}{w}\sum_{\mathrm{x=1}}^{w}\log_{a}\frac{exp\left[M_{j_{x}}^{N}i_{x}+h_{j_{x}}\right]}{\sum_{y=1}^{t}exp\left[M_{y}^{N}i_{x}+h_{y}\right]}, \end{array}$$

where *w* is the number of samples. *t* is the total number of categories, because this article needs to identify 7 kinds of facial features, so the value is 7. *i* is the input feature vector of the fully connected layer before classification. *h* is the offset amount. *M*_*j*_*x*__^*N*^*i*_*x*_+*h*_*j*_*x*__ represents the target determination that the predicted category is true in the output matrix of the xth sample fully connected layer.

#### 2.3.2. Interaction Mechanism

To capture the feature relationship between layers of different scales, this study uses hierarchical bilinear pooling across layers to integrate different convolutional layer features from the same network and different networks, and the layers that need to be fused are the last *3* convolutional layers (*Conv4_0, Conv4_1, and Conv4_2*) of different scale networks activated by the *PReLU* function, as shown in Table 3. *PReLU4_0_j,j* *=* *0,1,2*°. Thereinto, *j* is the number of network labels in the first few columns. *0* is *3×3* networks. *1* is *5×5* networks. *2* is *7×7* networks.

The bilinear confluence of different cross-layer features is now divided into the following three categories.

(1) Different hierarchical characteristics of the same network. The feature graphs of the last three convolutional layers of the three networks after the *PReLU* function are activated, and a total of 9 sets of bilinear features are obtained by interacting in pairs in the same network.
The bilinear feature evaluation expression for a specific interaction is as follows:
  (5) $$\begin{array}{c} \left(\text{PReLU}4\text{\_0\_0}*\text{PReLU}4\text{\_}1\text{\_0}+\text{PReLU4\_0\_0}*\text{PReLU4\_2\_0}+\text{PReLU}4\text{\_}1\text{\_0}*\text{PReLU}4\text{\_}2\text{\_0}\right)\\ +\left(\text{PReLU}4\text{\_0\_}1*\text{PReLU}4\text{\_}1\text{\_}1+\text{PReLU4\_0\_1}*\text{PReLU4\_2\_1}+\text{PReLU}4\text{\_}1\text{\_}1*\text{PReLU}4\text{\_}2\text{\_}1\right)\\ +\left(\text{PReLU}4\text{\_0\_}2*\text{PReLU}4\text{\_}1\text{\_}2+\text{PReLU4\_0\_2}*\text{PReLU4\_2\_2}+\text{PReLU}4\text{\_}1\text{\_}2*\text{PReLU}4\text{\_}2\text{\_}2\right). \end{array}$$
Figure 3 shows a schematic diagram of the interaction of different layers of features of the same network, wherein each column of features corresponds to the output characteristics of the last three convolutional layers of the *3×3, 5×5, and 7×7* networks after activation by the activation function, and each dotted wireframe represents a set of features that interact in pairs.
(2) Different hierarchical characteristics of different networks. Two restrictions have been added to make the features of different layers of different scale networks interact.
  (1) The last convolutional layer of each network must participate in the interaction. This is because, on the one hand, the current mainstream neural network classification model directly flattens the features extracted by the last layer of convolution into one-dimensional vectors, or first reduces the dimension through the global average pool, and then tiles into one-dimensional vector classification. On the other hand, the last layer of a neural network typically contains high-frequency and global feature information for the input image, suitable for classification.
  (2) There is a mutual exclusion in different layers of different networks. Different layers of different networks are used as a group, divided into 3 groups, and each group has 3 layers, two interactions, and a total of 9 sets of bilinear interaction features.
The bilinear feature evaluation expression for a specific interaction is as follows:
  (6) $$\begin{array}{c} \left(\text{PReLU}4\text{\_0\_0}*\text{PReLU}4\text{\_}2\text{\_}1+\text{PReLU4\_0\_0}*\text{PReLU4\_1\_2}+\text{PReLU}4\text{\_}2\text{\_}1*\text{PReLU}4\text{\_}1\text{\_}2\right)\\ +\left(\text{PReLU}4\text{\_}1\text{\_0}*\text{PReLU}4\text{\_0\_}1+\text{PReLU4\_1\_0}*\text{PReLU4\_2\_2}+\text{PReLU}4\text{\_0\_}1*\text{PReLU}4\text{\_}2\text{\_}2\right)\\ +\left(\text{PReLU}4\text{\_}2\text{\_0}*\text{PReLU}4\text{\_}1\text{\_}1+\text{PReLU4\_2\_0}*\text{PReLU4\_0\_2}+\text{PReLU}4\text{\_}1\text{\_}1*\text{PReLU}4\text{\_0\_}2\right). \end{array}$$
(3) Different networks have the same depth location characteristics. Taking the same depth layer as a group, it can be divided into 3 groups, and each group has 3 layers, two interactions, and a total of 9 sets of bilinear interaction features. The bilinear feature evaluation expression for a specific interaction is as follows:

(7) $$\begin{array}{c} \left(\text{PReLU}4\text{\_0\_0}*\text{PReLU}4\text{\_0\_}1+\text{PReLU4\_0\_0}*\text{PReLU4\_0\_2}+\text{PReLU}4\text{\_0\_}1*\text{PReLU}4\text{\_0\_}2\right)\\ +\left(\text{PReLU}4\text{\_}1\text{\_0}*\text{PReLU}4\text{\_}1\text{\_}1+\text{PReLU4\_1\_0}*\text{PReLU4\_1\_2}+\text{PReLU}4\text{\_}1\text{\_}1*\text{PReLU}4\text{\_}1\text{\_}2\right)\\ +\left(\text{PReLU}4\text{\_}2\text{\_0}*\text{PReLU}4\text{\_}2\text{\_}1+\text{PReLU4\_2\_0}*\text{PReLU4\_2\_2}+\text{PReLU}4\text{\_}2\text{\_}1*\text{PReLU}4\text{\_}2\text{\_}2\right). \end{array}$$

### 2.4. Multilayer Information Fusion

When the convolutional neural network propagates forward, high-frequency information is obtained by convolution layer by layer, and the features extracted by the last layer are input to the fully connected layer and classified. Filtering layer by layer will lose some low-frequency feature information, such as texture, edges, and other detail information, resulting in information that cannot be fully utilized. To obtain useful low-frequency information and improve the recognition rate of facial feature images, this method converts the activation value of the current convolutional layer output into a new activation value by deconvolution, fuses it layer by layer, reduces dimension layer by layer, and finally classifies it into a fully connected layer, as shown in Figure 4.

If the convolutional layer before pooling is recorded as one stage, the MHBP [16] network has 3 pooled layers at the same depth, so the volume can be integrated into 4 stages. The convolution in Figure 4 is a convolution of one stage of the MHBP network, with 6 convolutional layers in each of the first 3 phases and a total of 9 convolutional layers in the last phase. The characteristics of the multiconvolutional layer and the specific fusion process are as follows.

**Step 1 .**

The feature map activation values of the 9 convolutional layer outputs of the last stage *n* are reduced to the dimensionality of all the convolutional layer feature maps in the previous stage by *torch.cat* splicing, through *1×1* convolutional fusion, and the activation values are obtained by activating *BN* and *PReLU* functions. It is then entered into the deconvolution layer to obtain the feature map activation value.

**Step 2 .**

The activation values obtained in step *1* and the activation values of all convolutional layers in the previous stage *n-1* after stitching are combined to do additive fusion. After the fusion feature map *c×h×w* has a total of 2 branch operations, one branch obtains the compression feature map *c×1×1* through global average pooling, and the other branch continues to obtain the feature map *c×h×w* activation value through deconvolution. The purpose of dimensionality reduction is to reduce parameters and speed up network operation.

**Step 3 .**

Step *1* is performed once, step *2* is repeated twice, and you can get *3* sets of dimensionality reduction feature maps; after splicing and fusing, it is expanded into a one-dimensional vector and then a total of *32* *×* *6* *×* *3* *=* *576-*dimensional face feature vectors, and it added them to the full connection layer of the *MHBP* network and classified face features.

## 3. Experiments and Analysis

### 3.1. Simulation Environment and Parameter Settings

To verify the performance of the method, experiments are conducted on ORL, Yale, and AR databases, which contain interference variables such as lighting, expression, occlusion, and posture. The bin number of the histogram in the experiment is set to *256*. The chi-square distance matching recognition is used in ORL libraries and AR libraries, and histogram intersection distance matching recognition is used in Yale libraries. The performance comparison is selected with typical recognition algorithms such as PCA [1], LDA [2], LDN [3], CBP [4], CBFD [5], CA-LBFL [6], and LBP [7], where ORL and AR library experimental data are from the literature [17], and Yale library experimental data are from the literature [18]. The hardware device used in the experiment is Intel *I7-11800h, 32 GB of RAM*, and the simulation environment is *MATLAB R2019a.*

### 3.2. Consideration of Image Tile Size

Since in feature extraction, the image needs to be chunked to obtain the histogram of each subblock, too large or too small chunks will affect the recognition effect. To select the best tiles, the number of tiles is usually controlled within a certain range for comparative experiments to find the best way to tile under each database. In Figure 5, the horizontal axis represents the number of blocks; that is, *2×4* represents the number of column blocks and the number of row blocks is *2* and *4*, respectively, and the vertical axis represents the recognition rate. From the results of Figure 5, it can be seen that the selection of blocks under the ORL library is *2×4*, and the recognition rate is the highest. The more blocks under Yale, the higher the recognition rate, and the best effect is selected as *10×10*. The recognition rate is highest when the blocks are *24×15 and 8×5* under the AR lighting subset and the AR face subset, respectively. Under the AR occlusion A subset and the AR occlusion B subset, the recognition rate increases with the increase in the number of blocks, and the blocking method has a great impact on the result, and the selection of tiles is *24×15*, which has the best recognition effect.

### 3.3. Results and Analysis Based on ORL Databases

The ORL database was created by Olivetti Research Laboratory in Cambridge, UK, with a total of *400* images and *40* people. Each person had *10* face samples, mainly containing changes in posture, with a resolution of *112×92*, and the experiment chose to normalize to *96×96* resolution.

To ensure the accuracy of the experiment, each person in the experiment randomly selected *2 ∼ 6* pictures as training samples and the rest as test samples. The average of *10* experiments is taken as the experimental results, and the experimental results are shown in Table 4.

As can be seen from Table 4, the recognition rate of each algorithm gradually increases as the number of samples increases. The algorithm proposed in this study has the highest recognition rate under different numbers of training samples. The LDA algorithm only uses the edge response to find the edge feature and only uses the maximum and minimum values to correspond to the direction. The spatial information obtained is very limited, and the effect is general. Compared with PCA, LDA, LDN, CBP, CBFD, CA-LBFL, and LBP, the recognition rate of the algorithm was increased by *6.31* percentage points, *4.75* percentage points, *4.37* percentage points, *4.28* percentage points, *3.33* percentage points, *5.71* percentage points, and *2.84* percentage points. When the number of training samples is small, the improvement is significant. The changes caused by gestures in the ORL library are mainly reflected in the texture of the image. In this study, the algorithm extracts the main edge features based on the relative deviation of the edge response and the absolute deviation of the original grayscale space. Simultaneously, based on the maximum value of grayscale in each direction, independent gray structure information is extracted, which can better capture textures, higher recognition rate, and better performance than other similar methods that integrate multispace features.

### 3.4. Results and Analysis Based on Yale Database

The Yale face database was collected by Yale University and consisted of *165* images and *15* persons. Each person contains *11* pictures with a resolution of *100×100*, mainly including changes in lighting and posture.

There are many variables in the sample graph of the Yale database, such as lighting and small occlusions. In this experiment, *2∼5* of the pictures were randomly selected as the training samples, and the remaining ones were used as the test samples. The average of the results of the *10* experiments is also taken as the final result, and the experimental results are shown in Table 5.

When only *2* pictures were trained, most of the algorithms did not perform well, and the PCA method only had a recognition rate of *78.34%*. It does not distinguish between directional information and is difficult to extract stable facial features. LDA, LBP, and the proposed algorithm all grasp the number of directions corresponding to the maximum value to extract features. This extraction method is more stable than PCA and has better recognition performance. Compared with PCA, LDA, LDN, CBP, CBFD, CA-LBFL, and LBP, the proposed algorithm increased by *11.36* percentage points, *7.85* percentage points, *6.63* percentage points, *9.38* percentage points, *6.66* percentage points, *6.14* percentage points, and *2.63* percentage points, respectively, and the improvement effect was most significant. In addition, the proposed algorithm has achieved a higher recognition rate under the number of different training samples.

The CBP algorithm uses the tic-tac-toe neighborhood to expand the sampling range and extracts features using the maximum and secondary maximum edge response values, and the number of information increases. On the basis of PCA, the LDA algorithm captures the main edge information by distinguishing different edge response values and using the direction information corresponding to the maximum and minimum values, and the performance is better. The LDN method uses the edge response difference in adjacent points to distinguish between different directional information, but the gradient information is extracted less and the recognition rate is improved less. CBFD calculates the difference in the response of the upper edge of the center symmetry, and the deviation information reflected by this difference can reflect the general direction of the edge texture, which has a certain improvement, but the number of information is limited. CA-LBFL uses CBFD to extract the deviation information of the central symmetry direction and supplements the gradient information by the edge response difference in adjacent points. The LBP algorithm records the change information of the local area by making the difference between the original edge response value and the adjacent point edge response value, which is actually based on the relative difference value to record the information, saves the main information, and has a certain effect improvement. The proposed algorithm obtains the relative deviation based on the edge response and then uses the forward and backward differences in each direction to obtain the absolute deviation, and the information of two deviations complements each other in the gradient space, grasping the most important edge texture information. At the same time, the direction of the largest grayscale is recorded, and the gray level information independent of the gradient space is recorded. The information of two spatial features is independent of each other, which together improve the face information and show the best recognition effect.

### 3.5. Results and Analysis Based on AR Database

The AR database contains more than *4,000* images of *126* individuals [19] with image pixels of *120×165*. Each person has *26* pictures, collected at different times, and therefore contains changes in age. Each period contains *13* pictures, divided into four subsets: expression, lighting, occlusion *A*, and occlusion *B*, with various environmental changes. It is also one of the most extensive databases currently used to test face recognition. This article experimented with images of *50* men and *50* women, each containing *13* images from the same period. The experimental results are shown in Table 6.

As can be seen from Table 6, the recognition rate of the algorithm in this study under various subsets of AR libraries has been significantly improved. Under the subset of lighting and expressions, the algorithm will perform better if it can still extract the same stable features when the lighting and expression change. Most of the algorithms show a good recognition effect under these two subsets, since most algorithms record the direction information for the maximum or minimum value. This directional information tends to have better robustness, while the PCA algorithm treats information in all directions equally. Therefore, when the conditions change, the recognition performance is poor. Compared with the recognition rate of PCA, LDA, LDN, CBP, CBFD, CA-LBFL, and LBP under expression subset, the recognition rate of the algorithm in this study was increased by *3.34* percentage points, *2.67* percentage points, *2.34* percentage points, *3* percentage points, *2* percentage points, and *1.67* percentage points, respectively.

Compared with the illumination subset, the recognition rate of PCA, LDA, LDN, CBP, CBFD, CA-LBFL, and LBP increased by *7* percentage points, *3.33* percentage points, *5* percentage points, *4* percentage points, *2* percentage points, *2* percentage points, *2.67* percentage points, and *1.67* percentage points, respectively. Among the comparative algorithms, LBP, which mainly records gradient information, performed best. On the basis of enriching the gradient information through double deviation, the proposed algorithm further supplements the grayscale information independent of the gradient, and the features are more distinguishable, so the recognition rate is higher.

Under the AR occlusion subset, some key organs of the human face are obscured, and the available information is greatly reduced. If the algorithm does not provide sufficient information about the key areas without occlusion, the recognition performance will be greatly reduced. The A subset of AR occlusion is sunglasses occlusion, and the information in the eye area is greatly disturbed, and the recognition rate of PCA, LDA, LDN, and CBP methods is less than *95%*. Compared with the recognition rate of PCA, LDA, LDN, CBP, CBFD, and CA-LBFL algorithms, the recognition rate of *8* percentage points, *5.33* percentage points, *1* percentage point, and *0.33* percentage points was increased by *9.33* percentage points, *8* percentage points, *8* percentage points, and *8* percentage points, respectively. Under arbor-obscured *B* scarf interference, the image almost loses detail in the mouth area. Therefore, if the ability to restore the details of the half of the face is not enough, the recognition rate will be greatly reduced. It can be seen that the algorithm recognition rate of the comparison is already below *80%*. Compared with the recognition rate of PCA, LDA, LDN, CBP, CBFD, CA-LBFL, and LBP algorithms, the recognition rate of *25.66* percentage points, *30.66* percentage points, *19.33* percentage points, *22.66* percentage points, *22* percentage points, *22* percentage points, *19.33* percentage points, and *9.66* percentage points, respectively, increased, which is far better than similar algorithms. Compared with similar algorithms, this algorithm makes full use of the double deviation, extracts gradient features from different angles, and supplements grayscale features. The fused dual-space feature has a stronger ability to restore face details, so the recognition rate is still the highest when there is a wide range of occlusion interference, and the effect is significantly improved.

## 4. Conclusion

To further improve the performance of face recognition, three different scale networks are designed as the backbone networks for extracting face features through the convolutional neural network research for face recognition applications. The autonomous fusion of multiscale features of the backbone network is realized by adding a multiscale feature fusion module to the network. At the same time, a hierarchical bilinear pooling network is introduced to integrate the cross-layer face characteristics of the same network and different networks to obtain the delicate face feature attributes with differentiation. Also, a multilayer information fusion method is proposed. The experimental results indicate that compared with other methods, the multilayer feature fusion method can effectively use the lost information and improve the accuracy of face classification. The network based on multiscale bilinear pooling can capture face features with obvious recognition and improve the face recognition rate. The next step is to design a lightweight neural network. The model uses pyramid pooling to improve the fusion of multilayer features, which can obtain higher operational efficiency and better recognition effect.

## Figures and Tables

**Figure 1:** Multiscale hierarchical bilinear pooling network structure.

**Figure 2:** Multiscale attention interaction module.

**Figure 3:** Feature interaction between different layers of the same network.

**Figure 4:** Multilayer information fusion.

**Figure 5:** Results of the chunk experiment of each database.

**Table 1:** Parameter configuration of MHBP model 1.

Phase	Type	3 × 3 mesh	5 × 5 mesh	7 × 7 mesh	Output
1 phase	Conv1_0	3 × 3	5 × 5	7 × 7	48 × 48 × 32
	Conv1_1	3 × 3	5 × 5	7 × 7	48 × 48 × 32
	Maxpool1	(3, 2, 1)	(3, 2, 1)	(3, 2, 1)	24 × 24 × 32

2 phases	Conv2_0	3 × 3	5 × 5	7 × 7	24 × 24 × 32
	Conv2_1	3 × 3	5 × 5	7 × 7	24 × 24 × 32
	Maxpool2	(3, 2, 1)	(3, 2, 1)	(3, 2, 1)	12 × 12 × 32

3 phases	Conv3_0	3 × 3	5 × 5	7 × 7	12 × 12 × 32
	Conv3_1	3 × 3	5 × 5	7 × 7	12 × 12 × 32
	Maxpool3	(3, 2, 1)	(3, 2, 1)	(3, 2, 1)	6 × 6 × 32

4 phases	Conv4_0	3 × 3	5 × 5	7 × 7	6 × 6 × 32
	Conv4_1	3 × 3	5 × 5	7 × 7	6 × 6 × 32
	Conv4_2	3 × 3	5 × 5	7 × 7	6 × 6 × 32

**Table 2:** Parameter configuration of MHBP model 2.

Phase	Type	Layered bilinear pooling layer	Output
Classification of convergence	FC1	Input 512×18	1 × 1 × 1024
	FC2	Input 1×1×1024	1 × 1 × 512
	Output	Input 1×1×512	1 × 1 × 7

**Table 3:** Bilinear interaction layer list.

Convolution layer	3×3 mesh	5×5 mesh	7×7 mesh	Port number
Conv4_0	PReLU4_0_0	PReLU4_0_1	PReLU4_0_2	32
Conv4_1	PReLU4_1_0	PReLU4_1_1	PReLU4_1_2	32
Conv4_2	PReLU4_2_0	PReLU4_2_1	PReLU4_2_2	32

**Table 4:** Recognition rates of various algorithms under the ORL library.

Algorithm	The sample number of each class was randomly selected				
	2	3	4	5	6
PCA	82.9	89.68	92.91	93.77	95.2
LDA	86.42	91.24	94.44	96.12	97.51
LDN	86.62	91.62	95.23	96.32	97.8
CBP	86.77	91.71	95.18	96.3	97.82
CBFD	86.98	92.66	95.36	97.12	98.08
CA-LBFL	84.59	90.28	93.9	94.54	95.47
LBP	87.94	93.15	96.29	97.74	98.5
Proposed	92.58	95.99	97.3	98.27	99.42

**Table 5:** Recognition rates of various algorithms under the Yale library.

Algorithm	The sample number of each class was randomly selected			
	2	3	4	5
PCA	78.26	81.92	82.64	84.6
LDA	81.77	85.34	86.21	86.92
LDN	82.99	86.5	88.25	90.14
CBP	80.24	83.2	83.61	85.17
CBFD	82.96	85.34	87.82	88.36
CA-LBFL	83.48	87.34	88.4	89.48
LBP	86.99	91.42	93.3	94.02
Proposed	89.62	92.92	93.73	94.36

**Table 6:** Recognition rates of various algorithms under AR libraries.

Algorithm	AR expression	AR photoperiod	AR cover a	AR cover B
PCA	96.25	92.92	89.92	71.59
LDA	96.59	96.59	91.25	66.59
LDN	96.92	94.92	91.25	77.92
CBP	97.25	95.92	93.92	74.59
CBFD	96.59	97.92	98.25	75.25
CA-LBFL	97.59	97.25	98.92	77.92
LBP	97.92	98.25	99.25	87.59
Proposed	99.59	100	99.25	97.25

## Data Availability

The labeled dataset used to support the findings of this study is available from the corresponding author upon request.
